The article "The improvement of large High-Density Lipoprotein (HDL) particle levels, and presumably HDL metabolism, depend on effects of low-carbohydrate diet and weight loss" was retracted in 2016. Reasons: plagiarism; plagiarized data; content taken during peer review; overlap with other authors' work.

# The improvement of large High-Density Lipoprotein (HDL) particle levels, and presumably HDL metabolism, depend on effects of low-carbohydrate diet and weight loss

**DOI:** 10.17179/excli2015-642

**Published:** 2016-02-23

**Authors:** C. Finelli, P. Crispino, S. Gioia, N. La Sala, L. D'amico, M. La Grotta, O. Miro, D. Colarusso

**Affiliations:** 1 Center of Obesity and Eating Disorders, Stella Maris Mediterraneum Foundation, Chiaromonte, Potenza, Italy; 2 U.O.C. Medicina Interna, Urgenza ed Accettazione, P.O. S. Giovanni, Lagonegro - ASP Potenza

**Keywords:** obesity, HDL, low carbohydrate diet and weight loss

## Abstract

Depressed levels of atheroprotective large HDL particles are common in obesity and cardiovascular disease (CVD). Increases in large HDL particles are favourably associated with reduced CVD event risk and coronary plaque burden. The objective of the study is to compare the effectiveness of low-carbohydrate diets and weight loss for increasing blood levels of large HDL particles at 1 year. This study was performed by screening for body mass index (BMI) and metabolic syndrome in 160 consecutive subjects referred to our out-patient Metabolic Unit in South Italy. We administered dietary advice to four small groups rather than individually. A single team comprised of a dietitian and physician administered diet-specific advice to each group. Large HDL particles at baseline and 1 year were measured using two-dimensional gel electrophoresis. Dietary intake was assessed via 3-day diet records. Although 1-year weight loss did not differ between diet groups (mean 4.4 %), increases in large HDL particles paralleled the degree of carbohydrate restriction across the four diets (p<0.001 for trend). Regression analysis indicated that magnitude of carbohydrate restriction (percentage of calories as carbohydrate at 1 year) and weight loss were each independent predictors of 1-year increases in large HDL concentration. Changes in HDL cholesterol concentration were modestly correlated with changes in large HDL particle concentration (r=0.47, p=.001). In conclusion, reduction of excess dietary carbohydrate and body weight improved large HDL levels. Comparison trials with cardiovascular outcomes are needed to more fully evaluate these findings.

## Introduction

Cardiovascular disease (CVD) remains the leading cause of death throughout the world, and greater insight into the relative effects of various diets on CVD risk remains a public health priority (Eckel et al., 2014[7]; Jensen et al., 2014[15]).

New insights into the cardiovascular effects of diets inducing weight loss may be gained by measuring their effects on blood levels of large, fully matured, particles of high-density lipoprotein (HDL) (Rosenson et al., 2013[29]). Abnormally low levels of large HDL particles indicative of impaired HDL metabolism and atherogenic dyslipidaemia are common among overweight/obese patients with cardiovascular risk factors (Kouda, 2015[19]; Phillips and Perry, 2015[26]; Reina et al., 2015[27]; Samino et al., 2015[33]; Savolainen, 2015[35]). 

The article "The improvement of large High-Density Lipoprotein (HDL) particle levels, and presumably HDL metabolism, depend on effects of low-carbohydrate diet and weight loss" was retracted in 2016. Reasons: plagiarism; plagiarized data; content taken during peer review; overlap with other authors' work.

Increased levels of large HDL particles are potent predictors of reduced risk of CVD events, reduced atherosclerotic plaque burden, and longevity (Barzilai et al., 2003[2]; Filippatos and Elisaf, 2013[10]; Kim et al., 2014[17]; Russo et al., 2014[31]), whereas reduced levels of HDL cholesterol are potent predictors of metabolic syndrome (Finelli et al., 2006[11]; Savastano et al., 2015[34]; Tarantino et al., 2011[44]). Furthermore, centenarians and their offspring are known to have relatively high levels of large HDL particles (Barzilai et al., 2003[2]). Currently, available evidence supports the use of HDL particle number as the biomarker of choice to assess the contribution of HDL to cardiovascular risk, as reported by Rosenson et al. (2015[30]). Another, it is hypothesized, by Chyu and Shah, that in addition to HDL infusion therapy an alternative way to exploit beneficial cardiovascular effects of HDL/ApoA-1 is to use gene transfer (Chyu and Shah, 2015[4]). 

The aim of our study was to evaluate whether reduction of dietary carbohydrate and weight loss, resulted in clinically meaningful improvements in large HDL levels and presumably HDL metabolism, standard lipid profiles being inadequate for measuring such improvements. 

## Methods

### Patients

This study was performed screening 160 consecutive patients referred to our out-patient Metabolic Unit from South Italy. Patients 1-40 were assigned to the Atkins diet, patients 41-80 to the Zone diet, patients 81-120 to Weight Watchers diet, and patients 121-160 to the Ornish diet. We included only 93 patients, of any age with body mass index (BMI) between 27 and 42 kg/m^2^, having at least one of the following metabolic cardiac risk factors: fasting glucose > 110 mg/dl, total cholesterol > 200 mg/dl, low density lipoprotein (LDL) cholesterol > 130 mg/dl, high density lipoprotein (HDL) cholesterol < 40 mg/dl, triglycerides > 150 mg/dl, systolic blood pressure > 145 mmHg, diastolic blood pressure > 90 mmHg, or oral medication to treat hypertension, diabetes, or dyslipidaemia. Candidates (n=67) were excluded due to unstable chronic illness, insulin therapy, clinically significant abnormalities of liver, kidney or thyroid tests, weight loss medication, or pregnancy. The study was carried out according to the principles of the Declaration of Helsinki as revised in 2000 and written consent was obtained at the beginning of the study from each patient. Participants did not receive any monetary compensation. 

The article "The improvement of large High-Density Lipoprotein (HDL) particle levels, and presumably HDL metabolism, depend on effects of low-carbohydrate diet and weight loss" was retracted in 2016. Reasons: plagiarism; plagiarized data; content taken during peer review; overlap with other authors' work.

### Intervention

We administered dietary advice to small groups rather than individually. A single medical team comprised of a dietitian and physician nutritionist dispensed diet-specific advice to each group, meeting for one hour on four moments during the first two months of the study, as reported by Dansinger's study (Dansinger et al., 2005[5]). At the first meeting, the medical team communicated the diet attributed and specified the corresponding rationale and written materials. Following meetings attempted to maximize adherence by supporting positive dietary differences and addressing obstacles to adherence. The Atkins diet group attempted for less than 20 grams of carbohydrate day to day, with a progressive increase toward 50 grams day to day. The Zone group attempted for a 40-30-30 balance of percent calories from carbohydrate, fat, and protein, respectively. The Weight Watchers group attempted to keep total day-to-day “points” in a range regulated by current weight. Each “point” was approximately 50 calories, and most patients attempted for 24-32 points day to day. Lists produced by the Weight Watchers Corporation established point values of usual foods. The Ornish group attempted for a vegetarian diet containing 10 % of calories from fat. The benefit of these programs is that they are balanced nutritionally and, above all, that they provide precise information about the quantity of the individual nutrients. The reduction in calories makes people hungry and thus leads to discontinuation of the program.

In an effort to isolate the nutritional component of each plan, we standardized recommendations pertaining to supplements, physical activity, and external support, as reported by Dansinger's study (Dansinger et al., 2005[5]). We encouraged all patients to take a non-prescription multivitamin daily, obtain at least 60 minutes of physical activity weekly, and avoid commercial support services. To approximate the realistic long-term sustainability of each diet, we asked patients to follow their dietary assignment to the best of their ability until their two-month assessment, after which time we encouraged them to follow their assigned diet according to their own self-determined interest level, as reported by Dansinger's study (Dansinger et al., 2005[5]).

### Assessment of dietary intake and outcome measures

We asked participants to complete three-day food records at baseline, one, two, six, and 12 months (Schröder et al., 2001[37]). Utilizing a computerized diet analysis program (Nutritionist Five, version 2.3, First DataBank Inc.) we calculated the average day to day of each nutritional components (macro- and micro-nutrient) intakes.

The article "The improvement of large High-Density Lipoprotein (HDL) particle levels, and presumably HDL metabolism, depend on effects of low-carbohydrate diet and weight loss" was retracted in 2016. Reasons: plagiarism; plagiarized data; content taken during peer review; overlap with other authors' work.

We assessed clinical changes at baseline, two, six, and 12 months. Patients were blinded to the timing of the evaluations until two weeks prior to each visit, and the baseline measurement occurred within two weeks prior to the nutritional intervention. Study nurses and laboratory personnel were blinded to patients' dietary attribution. We determined body weight using a single calibrated scale (Detecto) while the patients were wearing light clothing and no shoes. We evaluated waist size as the average of two readings at the umbilicus utilizing a spring calibrated tape measure, and blood pressure as the average of one reading in each arm while sitting, using an automated instrument with digital readout (Dinamap, Critikon Inc.). Blood samples were drawn in fasting individuals. To have every laboratory test performed (serum lipids, glucose, insulin, and high sensitivity C-reactive protein), venous blood samples from the antecubital vein were obtained following standard procedures (Warnick, 2000[49]).

Total plasma apoA-I concentrations at baseline and 12 months were evaluated with a turbidimetric immunoassay (Wako Diagnostics) on a Hitachi 911 analyzer. ApoA-I-containing HDL subpopulations were determined by 2D non denaturing gel electrophoresis, immunoblotting, and image analysis as described by Asztalos et al. (2005[1]). All measurements were performed in our laboratory in the same way, and strict quality control procedures were followed. The interassay and intra-assay coefficients of variation were < 5 % for the lipid measurements and < 10 % for the apoA-I and HDL subpopulation determinations, as described by Asztalos et al. (2005[1]). All plasma samples were stored at −80 °C and were never thawed until analysis. The effects of long-term storage on HDL subspecies were evaluated, and no significant mutations in the values acquired after the valuation of the same samples fresh and from short-term and long-term storage were observed (Asztalos et al., 2005[1]).

### Statistical analysis

We used standard statistical software (SPSS version 17.0) to compute for each clinical and nutritional variable the means and standard deviations (SD) at baseline and one-year, the absolute and percent change from baseline, and one-sample t-tests to assess the null hypothesis of no change from baseline. Linear regression was used to calculate the p-value for linear trend for 1-year absolute change from baseline across the Atkins, Zone, Weight Watchers, and Ornish diets, respectively. Pearson correlation coefficients were used to assess the univariate associations between variables, and forward stepwise linear regression was used to evaluate the independent associations of nutritional and clinical (weight, waist size, and exercise) variables with large HDL levels. All p-values were two-sided; a value of < 0.05 was considered statistically significant.

The article "The improvement of large High-Density Lipoprotein (HDL) particle levels, and presumably HDL metabolism, depend on effects of low-carbohydrate diet and weight loss" was retracted in 2016. Reasons: plagiarism; plagiarized data; content taken during peer review; overlap with other authors' work.

## Results

Of 93 participants who completed the 1-year intervention, blood samples were available for analysis in 88 (n=20 in Atkins diet group; n=22 in Zone diet group; n=26 in Weight Watchers group; n=20 in Ornish diet group) cases (95 %). The mean age at baseline was 49 (SD=10) years, 43 (49 %) were male, and 67 (76 %) were Caucasian. For each diet group, absolute values at baseline and 1 year for relevant nutritional and biochemical cardiovascular risk variables are noted in Table 1(Tab. 1). Statistically significant macronutrient gradients (p < 0.05 for linear trend) across the four diets were present at 1 year for dietary carbohydrate, total fat, saturated fat, protein, fiber, and cholesterol.

The mean 1-year weight loss for all participants was 4.4 % (SD 6.3 %) with no statistical difference between diet groups (Figure 1a(Fig. 1)). In contrast, the mean increase in large HDL particles paralleled the degree of carbohydrate restriction recommended by each eating strategy (Figure 1b(Fig. 1)). At 1 year, large HDL particles were increased from baseline by 36 % for Atkins, 32 % for Zone, 16 % for Weight Watchers, and 2 % for Ornish (p < 0.001 for linear trend, Figure 2a(Fig. 2)). In comparison, HDL cholesterol increased approximately 16 % in the Atkins, Zone, and Weight Watchers groups and 1 % in the Ornish group at 1 year (Figure 2a(Fig. 2)). The univariate correlation between 12-month absolute change in HDL cholesterol versus absolute change in large HDL was less than 0.5 (Pearson r=0.47, p=0.001, Figure 2b(Fig. 2)).

Weight loss augmented the beneficial effect of carbohydrate restriction on large HDL levels (Figure 3a(Fig. 3)). When each of the four diet groups were pooled, percent weight loss (r=0.22, p=0.038) and reduced dietary carbohydrate intake (r=0.34, p=0.001) at 1 year were each predictive of increased levels of large HDL. This is illustrated in Figure 3(Fig. 3) according to clinically relevant categories of dietary carbohydrate intake (Figure 3b(Fig. 3)) and weight loss (Figure 3c(Fig. 3)).

In linear regression modelling, the strongest independent predictors of absolute changes in large HDL levels at 1 year were 1-year changes in dietary carbohydrate intake (as a proportion of calories, p < 0.001) and changes in body weight (percent weight loss, p=0.034). After accounting for these two factors (r=0.43, r2=0.19), the effects of 1-year changes in dietary intake of calories, sugars, protein, total fat, saturated fat, cholesterol, and fiber were each non-significant (p>0.05), as were changes in waist size and exercise. The 1-year level of large HDL (mg/dL) was closely predicted (r=0.84, r2=0.70, p<0.001) by accounting for the baseline level of large HDL along with the carbohydrate intake and weight loss. To further illustrate this relationship and facilitate clinical interpretation, Figure 4(Fig. 4) demonstrates predicted 1-year increases in large HDL.

The article "The improvement of large High-Density Lipoprotein (HDL) particle levels, and presumably HDL metabolism, depend on effects of low-carbohydrate diet and weight loss" was retracted in 2016. Reasons: plagiarism; plagiarized data; content taken during peer review; overlap with other authors' work.

## Discussion

We found that dietary carbohydrate restriction and weight loss were each independent predictors of improved blood levels of large protective HDL particles at 1 year. These particles have been shown to be the most effective in delivering cholesterol from the bloodstream back to the liver, enhancing reverse cholesterol transport (Zannis et al., 2006[50]). Individuals with CVD, obesity, type 2 diabetes and/or metabolic syndrome commonly have abnormal HDL metabolism (Filippatos and Elisaf, 2013[10]; Kim et al., 2014[17]; Rosenson et al., 2013[29]; Russo et al., 2014[31]), including reduced levels of large HDL, and our data strengthen the evidence that carbohydrate restriction and weight loss help normalize HDL metabolism and atherogenic dyslipidaemia (Lee et al., 2015[20]; Mascarenhas-Melo et al., 2013[23]; Tay et al. 2014[45]; Volek et al., 2009[48]; Zhang et al., 2015[51]). Relative improvements in large HDL levels were much more pronounced than improvements in HDL cholesterol levels, which were modest and not highly correlated with improvements in large HDL. Specifically measuring this cardiovascular risk factor unmasked a beneficial effect of carbohydrate restriction that was not previously visible with a standard lipid profile.

One plausible mechanism linking carbohydrate restriction and weight loss to improved HDL metabolism is via cholesteryl ester transfer protein (CETP). The activity of this enzyme, which transfers cholesteryl ester from HDL particles to LDL and VLDL particles in exchange for triglyceride, is known to be significantly increased in CVD and obesity and normalize in parallel with weight loss (Miller, 2015[25]; Scharnagl et al., 2014[36]). It is plausible that excess dietary intake of refined carbohydrates upregulates CETP activity, perhaps via postprandial and/or chronic elevations of glucose, insulin, triglyceride, and/or VLDL (Kontush et al., 2013[18]; Miller, 2015[25]; Scharnagl et al., 2014[36]; Sprandel et al. 2015[41]), and carbohydrate restriction plausibly reverses this hyperactivity, especially in the setting of insulin re-sistance and atherogenic dyslipidaemia. This hypothesized mechanism is compatible with other data showing that carbohydrate restriction and weight loss each improve levels of small dense LDL particles (Siri-Tarino et al., 2009[40]; Tay et al. 2014[45]; Volek et al., 2009[48]), and the strong correlation between improvements in large HDL and small-dense LDL particles is consistent with a common underlying mechanism (Mascarenhas-Melo et al., 2013[23]; Shoji et al., 2009[39]).

The article "The improvement of large High-Density Lipoprotein (HDL) particle levels, and presumably HDL metabolism, depend on effects of low-carbohydrate diet and weight loss" was retracted in 2016. Reasons: plagiarism; plagiarized data; content taken during peer review; overlap with other authors' work.

Our findings support the gathering notion that changes in HDL cholesterol levels may fail to adequately reflect beneficial or detrimental changes in HDL metabolism (Joshi et al., 2016[16]; Liu et al., 2015[21]; Madahian et al., 2014[22]; Rohatgi, 2015[28]; Schwendeman et al., 2015[38]). Normal HDL metabolism appears to be crucially important for a wide variety of physiological functions including reverse cholesterol transport and protection from cardiovascular disease (Joshi et al., 2016[16]; Liu et al., 2015[21]; Rohatgi, 2015[28]; Schwendeman et al., 2015[38]). Although levels of HDL cholesterol are clearly and consistently predictive of cardiovascular disease risk in epidemiological studies, some randomized trials of medications that raise HDL cholesterol levels (Elshazly et al., 2015[8]; Sacks et al., 2014[32]) and a negative Mendelian randomization study of plasma HDL cholesterol (Voight et al., 2012[47]) have highlighted the need to more fully understand the complex relationships between HDL, atherosclerosis, and CVD. More sophisticated measures of HDL metabolism, including HDL subfraction analysis, may potentially unmask previously overlooked relationships between improved HDL metabolism and improved cardiovascular outcomes.

Our findings highlight the need for comparative effectiveness trials of various eating strategies on actual cardiovascular event rates (Eckel et al., 2014[7]; Jensen et al., 2014[15]). Surrogate clinical markers, including next-generation blood markers of cardiovascular disease risk, are important but remain an inadequate replacement for determining actual clinical outcomes in dietary trials. Various eating strategies each have individual strengths and drawbacks making it impossible to know with certainty their actual net effects relative to one another on atherosclerosis, coronary plaque accumulation, rates of myocardial infarction, stroke, and longevity. For example, the Atkins diet was the best for restoring levels of large HDL in our trial, and this type of eating strategy has been strong for improving a wide variety of clinical markers (Hu et al., 2015[14]; Tay et al., 2015[46]), especially glycemic control and other cardiovascular risk markers in type 2 diabetes and metabolic syndrome (Feinman et al., 2015[9]). However, the Atkins diet liberalizes dietary saturated fat and animal protein, and simultaneously reduces fruit, vegetable, and fiber intake, potentially limiting or offsetting the potential health benefits of this strategy. Furthermore, compared to other eating strategies, an Atkins-style strategy could potentially adversely interact with the gut microbiota, for example via increased blood levels of trimethylamine-N-oxide (TMAO) induced by increased dietary choline and carnitine intake (Finelli and Tarantino, 2014[13]; Mente et al., 2015[24]), insulin resistance via increased artificial sweetener intake (Suez et al., 2014[42]), and/or adverse changes to the diversity and ecology of the gut microbiota (Chumpitazi et al. 2015[3]; Finelli et al., 2014[12]; Tarantino and Finelli, 2015[43]). Given so much remaining uncertainty raised by a diverse spectrum of diets, each with mixed known and unknown physiological effects, and by trials with surrogate outcomes, it is increasingly clear that actual outcomes trials are required to adequately assess the health effects of various clinically relevant eating strategies.

The article "The improvement of large High-Density Lipoprotein (HDL) particle levels, and presumably HDL metabolism, depend on effects of low-carbohydrate diet and weight loss" was retracted in 2016. Reasons: plagiarism; plagiarized data; content taken during peer review; overlap with other authors' work.

Our study has several important strengths and limitations. The data we present here come from a well-designed randomized trial of one year duration, however a limited number of patients (n=88) contributed to the data set, and we did not collect data beyond one year. The dietary intake data are based on 3-day diet records, which are a reasonably strong method for assessing dietary intake (Schröder et al., 2001[37]); however, the dietary data are based on self-reporting, and only reflect a snapshot of each individual's intake. The intervention was based on dietary advice, which corresponds to a clinically realistic intervention, however actually providing the food would have been advantageous for more clearly defining the effect of various diets on levels of large HDL particles. We used linear regression in an effort to disentangle the individual effects of dietary carbohydrate, protein, fat, saturated fat, cholesterol, and fiber, however this approach is susceptible to confounding and the dietary intervention was not designed to measure the individual effects of each macronutrient. Measuring large HDL levels via 2-dimensional electrophoresis is a highly accurate method for measuring large HDL particle levels (Dullens et al., 2007[6]; Rosenson et al., 2013[29]; Warnick, 2000[49]), however many clinicians are unfamiliar with the use of this technology in the clinical setting. Furthermore, although large HDL particles are more strongly predictive of cardiovascular disease prevention than HDL cholesterol levels, our study did not measure levels of HDL functionality, CETP activity, or lecithin-cholesterol acyltransferase (LCAT) activity, which may have added important insights (Kontush et al., 2013[18]; Miller, 2015[25]; Scharnagl et al., 2014[36]; Sprandel et al. 2015[41]).

The article "The improvement of large High-Density Lipoprotein (HDL) particle levels, and presumably HDL metabolism, depend on effects of low-carbohydrate diet and weight loss" was retracted in 2016. Reasons: plagiarism; plagiarized data; content taken during peer review; overlap with other authors' work.

In conclusion, we hypothesize that curbing dietary intake of refined carbohydrates decrease atherogenic dyslipidaemia, especially in the setting of insulin resistance. Dietary strategies that reduce refined sources of starch and sugar may potentially reduce cardiovascular disease and mitigate the epidemic of residual cardiovascular risk attributed to suboptimal eating patterns, however clinical trials with actual cardiovascular outcomes are required to properly address this public health concern.

## Disclosure statement

The authors declare that there are no conflicts of interest.

## Figures and Tables

**Table 1:** Baseline and one-year values for clinical variables in patients with 1-year data available for levels of large HDL*

**Figure 1:** a) Mean change in weight at 1 year according to diet type; b) Mean change in large HDL at 1 year according to diet type

**Figure 2:** a) Mean percent change in HDL cholesterol and large HDL at 1 year according to diet type; b) Absolute change in HDL cholesterol and large HDL at 1 year, scatterplot comparison

**Figure 3:** a) Mean change in large HDL at 1 year according to diet type, stratified by 1 year weight loss above vs. below the median; b) Mean change in large HDL at 1 year according to categories of dietary carbohydrate intake at 1 year; c) Mean change in large HDL at 1 year according to categories of percent weight loss at 1 year

**Figure 4:** Predicted increase in large HDL level at 1 year according to projected carbohydrate intake and weight loss

## References

[1] Asztalos BF, Collins D, Cupples LA, Demissie S, Horvath KV, Bloomfield HE (2005). Value of high-density lipoprotein (HDL) subpopulations in predicting recurrent cardiovascular events in the Veterans Affairs HDL Intervention Trial. Arterioscler Thromb Vasc Biol.

[2] Barzilai N, Atzmon G, Schechter C, Schaefer EJ, Cupples AL, Lipton R (2003). Unique lipoprotein phenotype and genotype associated with exceptional longevity. JAMA.

[3] Chumpitazi BP, Cope JL, Hollister EB, Tsai CM, McMeans AR, Luna RA (2015). Randomised clinical trial: gut microbiome biomarkers are associated with clinical response to a low FODMAP diet in children with the irritable bowel syndrome. Aliment Pharmacol Ther.

[4] Chyu KY, Shah PK (2015). HDL/ApoA-1 infusion and ApoA-1 gene therapy in atherosclerosis. Front Pharmacol.

[5] Dansinger ML, Gleason JA, Griffith JL, Selker HP, Schaefer EJ (2005). Comparison of the Atkins, Ornish, Weight Watchers, and Zone diets for weight loss and heart disease risk reduction: a randomized trial. JAMA.

The article "The improvement of large High-Density Lipoprotein (HDL) particle levels, and presumably HDL metabolism, depend on effects of low-carbohydrate diet and weight loss" was retracted in 2016. Reasons: plagiarism; plagiarized data; content taken during peer review; overlap with other authors' work.

[6] Dullens SP, Plat J, Mensink RP (2007). Increasing apoA-I production as a target for CHD risk reduction. Nutr Metab Cardiovasc Dis.

[7] Eckel RH, Jakicic JM, Ard JD, de Jesus JM, Houston Miller N, Hubbard VS (2014). 2013 AHA/ACC guideline on lifestyle management to reduce cardiovascular risk: a report of the American College of Cardiology/American Heart Association Task Force on Practice Guidelines. Circulation.

[8] Elshazly MB, Quispe R, Michos ED, Sniderman AD, Toth PP, Banach M (2015). Patient-level discordance in population percentiles of the total cholesterol to high-density lipoprotein cholesterol ratio in comparison with low-density lipoprotein cholesterol and non-high-density lipoprotein cholesterol: the very large database of lipids study (VLDL-2B). Circulation.

[9] Feinman RD, Pogozelski WK, Astrup A, Bernstein RK, Fine EJ, Westman EC (2015). Dietary carbohydrate restriction as the first approach in diabetes management: critical review and evidence base. Nutrition.

[10] Filippatos TD, Elisaf MS (2013). High density lipoprotein and cardiovascular diseases. World J Cardiol.

[11] Finelli C, Gallipoli P, Celentano E, Cacace G, Saldalamacchia G, De Caprio C (2006). Assessment of physical activity in an outpatient obesity clinic in southern Italy: results from a standardized questionnaire. Nutr Metab Cardiovasc Dis.

[12] Finelli C, Padula MC, Martelli G, Tarantino G (2014). Could the improvement of obesity-related co-morbidities depend on modified gut hormones secretion?. World J Gastroenterol.

[13] Finelli C, Tarantino G (2014). Non-alcoholic fatty liver disease, diet and gut microbiota. EXCLI J.

[14] Hu T, Yao L, Reynolds K, Whelton PK, Niu T, Li S (2015). The effects of a low-carbohydrate diet vs. a low-fat diet on novel cardiovascular risk factors: a randomized controlled trial. Nutrients.

[15] Jensen MD, Ryan DH, Apovian CM, Ard JD, Comuzzie AG, Donato KA (2014). 2013 AHA/ACC/TOS guideline for the management of overweight and obesity in adults: a report of the American College of Cardiology/American Heart Association Task Force on Practice Guidelines and The Obesity Society. J Am Coll Cardiol.

[16] Joshi PH, Toth PP, Lirette ST, Griswold ME, Massaro JM, Martin SS (2016). Association of high-density lipoprotein subclasses and incident coronary heart disease: The Jackson Heart and Framingham Offspring Cohort Studies. Eur J Prev Cardiol.

[17] Kim DS, Burt AA, Rosenthal EA, Ranchalis JE, Eintracht JF, Hatsukami TS (2014). HDL-3 is a superior predictor of carotid artery disease in a case-control cohort of 1725 participants. J Am Heart Assoc.

The article "The improvement of large High-Density Lipoprotein (HDL) particle levels, and presumably HDL metabolism, depend on effects of low-carbohydrate diet and weight loss" was retracted in 2016. Reasons: plagiarism; plagiarized data; content taken during peer review; overlap with other authors' work.

[18] Kontush A, Lhomme M, Chapman MJ (2013). Unraveling the complexities of the HDL lipidome. J Lipid Res.

[19] Kouda K, Nakamura H, Fujita Y, Hamada M, Kajita E, Nakatani Y (2015). HDL subclasses are heterogeneous in their associations with body fat, as measured by dual-energy X-ray absorptiometry: the Kitakata Kids Health Study. Clin Chim Acta.

[20] Lee JW, Kim EY, Yoo HM, Park CH, Song KY (2015). Changes of lipid profiles after radical gastrectomy in patients with gastric cancer. Lipids Health Dis.

[21] Liu X, Tao L, Cao K, Wang Z, Chen D, Guo J (2015). Association of high-density lipoprotein with development of metabolic syndrome components: a five-year follow-up in adults. BMC Public Health.

[22] Madahian S, Navab KD, Pourtabatabaei N, Seyedali S, Safar S, Vazirian S (2014). Inflammation, high density lipoprotein and endothelium. Curr Med Chem.

[23] Mascarenhas-Melo F, Sereno J, Teixeira-Lemos E, Marado D, Palavra F, Pinto R (2013). Implication of low HDL-c levels in patients with average LDL-c levels: a focus on oxidized LDL, large HDL subpopulation, and adiponectin. Mediators Inflamm.

[24] Mente A, Chalcraft K, Ak H, Davis AD, Lonn E, Miller R (2015). the relationship between trimethylamine-n-oxide and prevalent cardiovascular disease in a multiethnic population living in Canada. Can J Cardiol.

[25] Miller NE (2015). Cholesteryl ester transfer protein: ace of spades, queen of hearts, or the joker?. Front Pharmacol.

[26] Phillips CM, Perry IJ (2015). Lipoprotein particle subclass profiles among metabolically healthy and unhealthy obese and non-obese adults: Does size matter?. Atherosclerosis.

[27] Reina SA, Llabre MM, Allison MA, Wilkins JT, Mendez AJ, Arnan MK (2015). HDL cholesterol and stroke risk: The Multi-Ethnic Study of Atherosclerosis. Atherosclerosis.

[28] Rohatgi A (2015). High-density lipoprotein function measurement in human studies: focus on cholesterol efflux capacity. Prog Cardiovasc Dis.

[29] Rosenson RS, Brewer HB, Ansell B, Barter P, Chapman MJ, Heinecke JW (2013). Translation of high-density lipoprotein function into clinical practice: current prospects and future challenges. Circulation.

[30] Rosenson RS, Davidson MH, Le NA, Burkle J, Pourfarzib R (2015). Underappreciated opportunities for high-density lipoprotein particles in risk stratification and potential targets of therapy. Cardiovasc Drugs Ther.

[31] Russo GT, Giandalia A, Romeo EL, Alibrandi A, Horvath KV, Asztalos BF (2014). Markers of systemic inflammation and apo-ai containing hdl subpopulations in women with and without diabetes. Int J Endocrinol.

[32] Sacks FM, Carey VJ, Anderson CA, Miller ER, Copeland T, Charleston J (2014). Effects of high vs low glycemic index of dietary carbohydrate on cardiovascular disease risk factors and insulin sensitivity: the OmniCarb randomized clinical trial. JAMA.

The article "The improvement of large High-Density Lipoprotein (HDL) particle levels, and presumably HDL metabolism, depend on effects of low-carbohydrate diet and weight loss" was retracted in 2016. Reasons: plagiarism; plagiarized data; content taken during peer review; overlap with other authors' work.

[33] Samino S, Vinaixa M, Díaz M, Beltran A, Rodríguez MA, Mallol R (2015). Metabolomics reveals impaired maturation of HDL particles in adolescents with hyperinsulinaemic androgen excess. Sci Rep.

[34] Savastano S, Di Somma C, Colao A, Barrea L, Orio F, Finelli C (2015). Preliminary data on the relationship between circulating levels of Sirtuin 4, anthropometric and metabolic parameters in obese subjects according to growth hormone/insulin-like growth factor-1 status. Growth Horm IGF Res.

[35] Savolainen MJ (2015). Epidemiology: disease associations and modulators of HDL-related biomarkers. Handb Exp Pharmacol.

[36] Scharnagl H, Heuschneider C, Sailer S, Kleber ME, März W, Ritsch A (2014). Decreased cholesterol efflux capacity in patients with low cholesteryl ester transfer protein plasma levels. Eur J Clin Invest.

[37] Schröder H, Covas MI, Marrugat J, Vila J, Pena A, Alcántara M (2001). Use of a three-day estimated food record, a 72-hour recall and a food-frequency questionnaire for dietary assessment in a Mediterranean Spanish population. Clin Nutr.

[38] Schwendeman A, Sviridov DO, Yuan W, Guo Y, Morin EE, Yuan Y (2015). The effect of phospholipid composition of reconstituted HDL on its cholesterol efflux and anti-inflammatory properties. J Lipid Res.

[39] Shoji T, Hatsuda S, Tsuchikura S, Shinohara K, Kimoto E, Koyama H (2009). Small dense low-density lipoprotein cholesterol concentration and carotid atherosclerosis. Atherosclerosis.

[40] Siri-Tarino PW, Williams PT, Fernstrom HS, Rawlings RS, Krauss RM (2009). Reversal of small, dense LDL subclass phenotype by normalization of adiposity. Obesity (Silver Spring).

[41] Sprandel MC, Hueb WA, Segre A, Ramires JA, Kalil-Filho R, Maranhão RC (2015). Alterations in lipid transfers to HDL associated with the presence of coronary artery disease in patients with type 2 diabetes mellitus. Cardiovasc Diabetol.

[42] Suez J, Korem T, Zeevi D, Zilberman-Schapira G, Thaiss CA, Maza O (2014). Artificial sweeteners induce glucose intolerance by altering the gut microbiota. Nature.

[43] Tarantino G, Finelli C (2015). Systematic review on intervention with prebiotics/probiotics in patients with obesity-related nonalcoholic fatty liver disease. Future Microbiol.

[44] Tarantino G, Scopacasa F, Colao A, Capone D, Tarantino M, Grimaldi E (2011). Serum Bcl-2 concentrations in overweight-obese subjects with nonalcoholic fatty liver disease. World J Gastroenterol.

[45] Tay J, Luscombe-Marsh ND, Thompson CH, Noakes M, Buckley JD, Wittert GA (2014). A very low-carbohydrate, low-saturated fat diet for type 2 diabetes management: a randomized trial. Diabetes Care.

The article "The improvement of large High-Density Lipoprotein (HDL) particle levels, and presumably HDL metabolism, depend on effects of low-carbohydrate diet and weight loss" was retracted in 2016. Reasons: plagiarism; plagiarized data; content taken during peer review; overlap with other authors' work.

[46] Tay J, Luscombe-Marsh ND, Thompson CH, Noakes M, Buckley JD, Wittert GA (2015). Comparison of low- and high-carbohydrate diets for type 2 diabetes management: a randomized trial. Am J Clin Nutr.

[47] Voight BF, Peloso GM, Orho-Melander M, Frikke-Schmidt R, Barbalic M, Jensen MK (2012). Plasma HDL cholesterol and risk of myocardial infarction: a mendelian randomisation study. Lancet.

[48] Volek JS, Ballard KD, Silvestre R, Judelson DA, Quann EE, Forsythe CE (2009). Effects of dietary carbohydrate restriction versus low-fat diet on flow-mediated dilation. Metabolism.

[49] Warnick GR (2000). Measurement of cholesterol and other lipoprotein constituents in the clinical laboratory. Clin Chem Lab Med.

[50] Zannis VI, Chroni A, Krieger M (2006). Role of apoA-I, ABCA1, LCAT, and SR-BI in the biogenesis of HDL. J Mol Med (Berl).

[51] Zhang C, Gao F, Luo H, Zhang CT, Zhang R (2015). Differential response in levels of high-density lipoprotein cholesterol to one-year metformin treatment in prediabetic patients by race/ethnicity. Cardiovasc Diabetol.

